The article "Efficacy of Moxibustion in the Treatment of Parkinson's Disease Based on Meta-Analysis under Intelligent Medical Treatment" was retracted in 2023. Reasons: signs of a paper mill; suspected computer-generated content; unreliable results or conclusions; concerns about the data.

# Efficacy of Moxibustion in the Treatment of Parkinson's Disease Based on Meta-Analysis under Intelligent Medical Treatment

**DOI:** 10.1155/2022/8168152

**Published:** 2022-04-30

**Authors:** Qianqian Niu, Weijie Xu

**Affiliations:** ^1^Seven Department of Acupuncture and Moxibustion, Heilongjiang Academy of Traditional Chinese Medicine, Harbin, 150036 Heilongjiang, China; ^2^Kunming Health Vocational College, Kunming, 650000 Yunnan, China

## Abstract

Dementia in Parkinson's disease (PD) has become a major factor affecting the quality of life of patients with Parkinson's disease. Early detection and timely prevention can delay the progression of dementia, improve the quality of life of patients, and reduce the burden on society. This article is aimed at studying how to analyze the efficacy of moxibustion in the treatment of Parkinson's disease through meta-analysis on the basis of smart medicine. This article puts forward the related conceptual knowledge of smart medicine and meta-analysis and moxibustion treatment and proposes a deep learning method based on smart medicine to analyze the effects of moxibustion treatment on patients. The experiment in this article can be seen from the data in one of the figures that the highest curative effect of using a single moxibustion to treat Parkinson's disease is about 46%, while the curative effect of using a combination of moxibustion and Western medicine has reached 90%. It can be seen that a single moxibustion is not as effective as a combination of the two for Parkinson's disease. From the data in one of the tables, it can be seen that the proportion of Parkinson's disease in 2016 was 15%, showing an increase of 5%. By 2020, the proportion of Parkinson's disease was as high as 38%, and the growth rate reached 9%. It can be seen that the prevalence of this disease is getting higher and higher. Parkinson's disease has caused many undesirable effects on patients, such as slow movement, mental disorders, and a decline in mental state. Therefore, it is urgent to study the treatment of Parkinson's disease. Moxibustion can improve the patient's blood circulation and help the patient's local limbs to recover more easily and can help improve the patient's motor function.

## 1. Introduction

In recent years, the Internet of Things has gradually become the mainstream. The Internet of Things refers to the real-time collection of required information through sensors and other related equipment. With the development of Internet of Things-related technologies, the application and practice of Internet of Things technology in medical treatment has also attracted much attention. Smart medicine uses the Internet of Things technology to integrate medical-related resource information and forms a huge platform through network sharing for sharing medical information. Parkinson's disease (PD), also known as tremor palsy, is a common degenerative disease of the nervous system in middle-aged and elderly people. The main lesions are in the substantia nigra and striatum. Tremor, muscle rigidity, and decreased movement are the main clinical features of this disease. Parkinson's disease is the fourth most common neurodegenerative disease in the elderly [1, 2].

The intelligent medical equipment of the intelligent medical system can replace many traditional manual operations [3, 4]. Because of its low error rate and high efficiency, it can improve the hospital's resource allocation efficiency and reduce resource waste. In the intelligent nursing alarm system, the intelligent alarm can monitor the patient's health status in real time. After the patient has an abnormal state, an alarm will be generated, which can improve the work efficiency of medical staff.

The innovations of this article are as follows: (1) It introduces the related theoretical knowledge of smart medicine and meta-analysis and uses deep learning technology based on smart medicine to analyze how to treat Parkinson's moxibustion based on smart medicine and meta-analysis. (2) Based on the deep learning algorithm of intelligent medical treatment, the experiment and analysis of the effect of moxibustion in the treatment of Parkinson's disease are carried out. Through investigation and analysis, it is found that the use of moxibustion in the treatment of Parkinson's disease is of great significance.

## 2. Related Work

With the development of the society in recent years, smart medical care has also attracted more and more attention. Falup-Pecurariu and Diaconu believe that Parkinson's disease (PD) not only affects patients' sleep but also severely affects their quality of life. Their research shows that more than half of PD patients have sleep disorders. He used specific scales in the research to help screen and evaluate sleep dysfunction. However, the scholars did not reveal their research process, and the authenticity of the research conclusions is doubtful [5]. Sulzer et al. found that Parkinson's disease is related to alleles of the major histocompatibility complex. He used a set of defined peptides as the subject of his experiment. These peptides are derived from nucleoprotein, a protein that aggregates in Parkinson's disease. He explained the relationship between Parkinson's disease and specific major histocompatibility complex alleles. Although the scholar described the experimental subjects very clearly, he did not draw specific conclusions and did not explain the relationship between the two [6]. Jiang and Dickson found that Parkinson's disease (PD) is a chronic movement disorder in adults. He also found that in the past few decades, rodent models of PD using genetic strategies have been widely used to study the pathogenesis and treatment of PD. However, the scholars did not specify how to apply the PD rodent model to study the pathogenesis and treatment of PD [7]. Tarakad and Jankovic found that despite many efforts to determine specific and sensitive biomarkers, the diagnosis of Parkinson's disease (PD) is still based on clinical criteria, including the presence of basic motor characteristics, a combination of other motor characteristics, and many nonmotor characteristics. They found that dopamine agonists also play an important role as monotherapy in the adjuvant treatment of mild or moderately advanced disease. Although the scholars listed specific methods, they did not introduce how the method can be applied to mild or moderately advanced PD [8]. Chen et al. analyzed China's “One Belt One Road” initiative and “One Belt One Road” Chinese medicine development plan and discussed the measures of government agencies, academic groups, medical institutions, and other subjects. He comprehensively investigated various factors and put forward several suggestions on the development of moxibustion in China under the background of the “Belt and Road Initiative.” However, the scholars did not introduce what the few suggestions they wanted to make and did not draw specific conclusions [9]. Liu et al. explored the correlation between moxibustion and the distance of moxa sticks to provide clinical reference. He recorded the occurrence and frequency of moxibustion at distances of 5 cm, 4 cm, 3 cm, and 2 cm and finally found that the distance of 3 cm was the most comfortable distance for mild moxibustion. Although the scholars came to a conclusion and discussed the comfort of moxibustion at different distances, there is no reference data, which reduces the reliability of the experiment [10]. Bonvento found that in the era of ubiquitous smartphones and wireless networks, there are some applications that allow users to contact doctors, replenish prescriptions, and perform treatments with a simple click of a button. Today, people can use remote intelligent medical and video conferencing systems to talk to doctors in real time. This system enables patients to communicate their symptoms with doctors in time, reducing the pressure on doctors. And for the patient, it saves a lot of time and provides great convenience for the patient. However, the scholar did not cite specific examples to illustrate how smart medicine can bring convenience to people [11]. Liu et al. found that acupuncture, as an intervention of Chinese medicine, is widely used in clinical practice around the world. But there are still many problems. Although the scholars found many problems in the application of moxibustion, they did not specify the problems, and they have not proposed corresponding solutions [12]. Through the experimental analysis of scholars, we can see that moxibustion has been widely used in medicine and in people's daily life, and its effect on people is increasing. In daily medicine, people are also inseparable to smart medicine.

## 3. Basic Concepts of Smart Medicine and Moxibustion

The preclinical treatment for PD patients is mainly to relieve the clinical symptoms of PD patients and not control the progress of PD patients. Many researchers hope to control the disease of PD patients at the pathological level through certain treatment methods but only use Western medicine, which suggests difficulty in achieving a good therapeutic effect [13]. The symptoms of PD patients are shown in Figure 1.

As shown in Figure 1, the symptoms of PD patients mainly include slow movement, mental disorders, and the possibility of Alzheimer's [14]. You cannot take care of yourself in daily life, stand up after sitting down, turn over when lying in bed, untie shoelaces and buttons, put on shoes and socks or pants, shave, wash your face, and brush your teeth. Repeated exercise easily causes fatigue.

Smart medical and health services are the basis for ensuring human safety, quality of life and overall development, a necessary condition for supporting the sustainable development of human society and economy, and the basis for national development [15]. The structure of the intelligent medical system is shown in Figure 2.

As shown in Figure 2, smart medicine not only has an impact on smart diagnosis, smart care, health management, and medical management but, more importantly, smart medicine can also promote the development of precision medicine [16, 17].

Moxibustion has a good effect on the regulation of human body functions. The method of moxibustion is simple and safe and has no side effects on the human body, so it has attracted much attention. According to research, moxibustion can greatly improve the body's immune system and regulate endocrine [18]. The application of moxibustion is shown in Figure 3.

As shown in Figure 3, clinically, moxibustion can treat many diseases. However, during the burning process of moxibustion, a large amount of smoke is not only produced, which makes the medical environment worse, but it is also inefficient and inconvenient to operate. Therefore, the development of moxibustion has been greatly restricted.

The multifunctional intelligent moxibustion device is a comprehensive computer technology, sensor technology, invented based on the previous principles of moxibustion, and also combines the latest electronic computer technology and magnetic therapy [19]. The invention and universal application of intelligent moxibustion instruments have completely ended the development history of traditional moxibustion therapy that has burned for more than five thousand years. Using moxibustion therapy to prevent and treat diseases provides a safe, reliable, convenient, and fast modern intelligent moxibustion tool. The multifunctional intelligent moxibustion device is shown in Figure 4.

As shown in Figure 4, when the dedicated moxibustion device is heated, the patient's skin will also be heated and the sweat glands will relax. Therefore, the effective ingredients and volatile substances of moxibustion will quickly pass through the acupoints and meridians and directly act on the lesions [20], so as to achieve the purpose of preventive treatment.

A meta-analysis is a statistical analysis method that collects data and analyzes the results of multiple independent studies and uses the average effect size to answer research questions. It can be applied to evidence-based medicine and other scientific fields [21]. A meta-analysis is an important means of objectively synthesizing and analyzing data. It provides a summary for scientific research and guides the next research direction. The system structure diagram of a meta-analysis is shown in Figure 5.

As shown in Figure 5, compared with a single study, a meta-analysis can more accurately estimate the effects of medical treatment and health care by integrating all relevant studies, which helps to investigate the consistency and differences of various research evidence. For a small sample of clinical experimental research, a meta-analysis can calculate the accuracy of the power and effect size estimation. Therefore, a rationally designed and rigorous meta-analysis article can make a more objective evaluation of the evidence.

## 4. Deep Learning Method Based on Intelligent Medical Care

Deep learning is to learn the inherent laws and representation levels of sample data. The information obtained in the learning process is of great help to the interpretation of data such as text, images, and sounds. Its ultimate goal is to make machines have the ability to analyze and learn like humans and can recognize data such as text, images, and sounds. Some of the main results of deep learning appear in the field of computer vision. The field of vision mainly studies the understanding of images and videos and completes tasks such as target classification, detection, and segmentation. These are very useful for judging whether the patient's X-ray pictures contain malignant tumors. Convolutional neural networks are used to process spatially invariant data, which is an important technology in this field [22]. The deep learning structure diagram is shown in Figure 6.

As shown in Figure 6, deep learning is a very popular method in machine learning, covering multiple theoretical viewpoints. In order to achieve a more intelligent human-computer interaction, researchers imitated human brain and thinking and established various neural network models, and deep learning is one of them [23]. Deep learning is a multilevel representation learning method, through the creation of models to learn data characteristics and find better data.

### 4.1. Convolutional Neural Network

Convolutional neural network is a kind of feedforward neural network that contains convolution calculation and has a deep structure. It is one of the representative algorithms of deep learning. Convolutional neural network has the ability to characterize learning and can classify input information according to its hierarchical structure with translation invariance, so it is also called translation invariant artificial neural network. The convolutional layer performs convolution processing on the target image through the convolution kernel, generates a feature map, and realizes local feature perception and feature extraction. The convolutional neural network is shown in Figure 7.

As shown in Figure 7, the convolutional neural network is a multilayer network structure and is composed of multiple parts in series, mainly including a convolutional layer, a pooled sampling layer, and a fully connected layer.

The training of convolutional neural networks is supervised training. The general process of parameter training is as follows: inputting data, forwarding propagation layer by layer, and getting the network output of each layer; according to the difference between the actual output of the network and the expected output, use the BP algorithm to adjust the error in reverse and update the network parameters [24]. The training process of the fully connected layer mainly includes calculation output, back propagation, and weight update.

In the calculation output for layer l of the fully connected layer, the output result is formula (1):

(1) $$\begin{array}{c} u^{l}=W^{l}a^{l-1}+b, \end{array}$$

where *W*^*l*^ and *b* are weights and biases, respectively, *a*^*l*−1^ is the Sigmoid activation function, and the output range of this function is [0,1].

Assuming that *n* is the current sample number, the error *E*^*n*^ of the *n*-th sample is formula (2):

(2) $$\begin{array}{c} E^{n}=\frac{1}{2}\overset{c}{\underset{k=1}{\sum }}{\left(t_{k}^{n}-b_{k}^{n}\right)}^{2}=\frac{1}{2}{\left\|t^{n}-b^{n}\right\|}^{2}. \end{array}$$

In the formula, *t*^*n*^ is the expected output value of the *n*-th sample and *b*_*k*_^*n*^ represents the actual output value of the *n*-th sample through the network operation.

#### 4.1.1. Backpropagation

The backpropagation algorithm, referred to as BP algorithm, is a learning algorithm suitable for multilayer neural networks, which is based on the gradient descent method. The data is calculated through the layers of the network, and the error between the actual output and the expected output is obtained, which can be regarded as the sensitivity of the neuron [14]. The formula is formula (3):

(3) $$\begin{array}{c} \frac{\partial E}{\partial b}=\frac{\partial E}{\partial u}\frac{\partial u}{\partial b}. \end{array}$$

The formula for the sensitivity of the *δ*^*t*^ layer in the back propagation phase is formula (4):

(4) $$\begin{array}{c} \delta^{t}={\left(w^{l+1}\right)}^{T}\delta^{t+1}. \end{array}$$

Through the calculation of formula (4), the gradient of the given feature map is obtained, and formula (4) shows that the gradient of the bias basis is obtained by calculating the sum of the sensitivity of the feature map nodes in layer 1 [25].

Furthermore, downsampling is pooling. The sampling layer is implemented using related technologies. The purpose is to reduce the dimension of features and retain effective information, to a certain extent to avoid over-fitting. The function of the pooling sampling layer is to pool the feature maps. Therefore, the number of input and output feature maps is not changed, and the size of the feature maps has changed. The pooling process is as shown in formula (5):

(5) $$\begin{array}{c} a_{j}^{l}=f\left(\beta_{j}^{t}\text{down}\left(a_{j}^{l-1}\right)+b_{j}^{l}\right). \end{array}$$

Among them, down(*a*_*j*_^*l*−1^) is the pooling function and *β* and *b* represent the weight and bias, respectively.

The sensitivity calculation formula is formula (6):

(6) $$\begin{array}{c} \delta_{j}^{l}=f\left(u_{j}^{l}\right)*conv2{\left(\delta_{j}^{l+1}\right)}^{2}. \end{array}$$

The calculation of the bias *f*(*u*_*j*_^*l*^) in the pooling sampling layer is the same as the calculation of the bias in the convolutional layer.

### 4.2. Restricted Boltzmann Machine (RBM)

Restricted Boltzmann machine (RBM) is a kind of randomly generated neural network that can learn probability distribution through input data set. Restricted Boltzmann machine is an energy model. The network energy function *H*(*v*, *h*) of RBM is related to the visible layer, the hidden layer, and the parameters of each layer [26] (formula (7)):

(7) $$\begin{array}{c} H\left(v,h\right)=-\underset{i\in v}{\sum }a_{i}v_{i}-\underset{j\in h}{\sum }b_{j}h_{j}. \end{array}$$

In the formula, *a*_*i*_ and *a*_*i*_ are the parameter values of RBM and (*v*, *h*) is the connection weight between the visible layer node *i* and the hidden layer node *j*. The energy function formula of the RBM network defined by formula (7) can be calculated as the joint probability distribution of state (*v*, *h*) as formula (8):

(8) $$\begin{array}{c} P\left(v,h\right)=\frac{1}{Z}\exp\left(-H\left(v,h\right)\right). \end{array}$$

In the formula, *Z* is the normalization factor. Normalization is a way to simplify calculations; that is, a dimensional expression will be transformed into a dimensionless expression and become a scalar. This method is often used in a variety of calculations. From the joint probability distribution *P*(*v*, *h*), the node state of a certain layer can be obtained, and the conditional distribution of the state of the other layer is Equation (9):

(9) $$\begin{array}{c} P\left(v\left|h\right.\right)=\sigma \left(w_{ij}h_{j}+a_{i}\right). \end{array}$$

In the formula, *σ*(.) is the Sigmoid function and its general formula is (*w*_*ij*_*h*_*j*_ + *a*_*i*_). If the probability distribution *P*(*v*) of the observation data *v* is larger, the obtained network model has a stronger ability to restore the observation data [27]. The specific process of obtaining the probability distribution *P*(*v*) is formula (10):

(10) $$\begin{array}{c} P\left(v\right)=\underset{h}{\sum }P\left(v,h\right)=\frac{1}{z}\underset{h}{\sum }\exp\left(-H\left(v,h\right)\right). \end{array}$$

The likelihood function of the parameter *θ* ∈ {*w*, *a*, *b*} of the input data *v* is the selected probability distribution *P*(*v*). Adjust the parameter *θ*, as formula (11):

(11) $$\begin{array}{c} \theta^{\cdot }=\theta +\eta \frac{\partial InP\left(v\right)}{\partial \theta }. \end{array}$$

In the formula, the parameter *θ* ∈ {*w*, *a*, *b*} is expressed as the learning rate. At the same time, this article only considers the condition that the interlayer connection weight *w*_*ij*_ is regarded as a parameter. Through algebraic transformation, the result obtained is equation (12):

(12) $$\begin{array}{c} \frac{\partial InP\left(V\right)}{\partial W_{ij}}=-\underset{n}{\sum }P\left(h\left|v\right.\right). \end{array}$$

Among them, *v* is an arbitrary sample and *∂W*_*ij*_ is a specific training sample. Since *v* is related to *Z*, it is difficult to obtain the joint probability distribution *P*(*h*|*v*).

### 4.3. Improved Deep Belief Network

The deep belief network is composed of multilayer Boltzmann machines, and the Monte Carlo method is used in the network learning process. The deep belief network is a commonly used deep learning algorithm, and the deep belief network is fine-tuned through the BP neural network during the training process. BP neural network has solved many problems in artificial neural network algorithms since it was put forward, and it has been widely used. As researchers continue to discuss, the BP neural network has formed a more mature theoretical system, but the BP neural network is basically a gradient descent algorithm. In other words, it can only adjust down the slope and it is difficult to climb the slope. However, there are some shortcomings.

Artificial bee colony algorithm is an intelligent algorithm that imitates the honey-collecting behavior of bees and abstracts it as a mathematical model to solve multidimensional and multimode optimization problems. Because bees collect nectar and find nectar sources have global and certain randomness, artificial bee colony algorithm is an algorithm with global characteristics.

Suppose that the problem of dimension D is required to be solved. When the number of iterations is *t*, the spatial position of the nectar *i* is rand(0, 1), where *t* is the number of iterations at this time and *a*_*i*_^*t*^ and *L*_*d*_ are the upper and lower limits of the search space, respectively, such as formula (13),

(13) $$\begin{array}{c} a_{id}=L_{d}+\mathrm{rand}\left(0,1\right)\left(u_{d}-l_{d}\right), \end{array}$$

which means that the scout bee randomly selects one-dimensional search; *j* ∈ 1, 2, ⋯, *n* means randomly generating a nectar source different from *i* among NP nectar sources; *l*_*d*_ means affecting the perturbation amplitude.

When the new nectar source *V*_*i*_ = *v*_1_, *v*_2_, ⋯, *v*_*n*_ fitness value is greater than *a*_*I*_, the greedy selection method *V*_*i*_ is used to replace *V*_*i*_, and vice versa. After all reconnaissance bees complete the calculation of formula (13), they fly back to the hive to share the nectar source information. The observation bee based on the information shared by the hired bee is in formula (14):

(14) $$\begin{array}{c} p_{i}={\text{fit}}_{i}/\overset{np}{\underset{i=1}{\sum }}{\text{fit}}_{i}. \end{array}$$

This section fully considers the characteristics of the fine-tuning part of the deep belief network training process. Based on the research of artificial bee colony algorithm and BP neural network, a method based on artificial bee colony algorithm and deep belief network is proposed.

Here, the artificial bee colony algorithm optimization method can also be used to check whether the BP neural network falls into a local minimum. If the adjusted structure of the BP algorithm is already near the global minimum, then the search results of the artificial bee colony algorithm are ineffective. At this time, the artificial bee colony algorithm only plays a discriminating role; if the BP algorithm adjusts the structure at the local extreme point, then the global search of the artificial bee colony algorithm can jump out of this local extreme point and search for the best point.

### 4.4. Cost Function

The cost function is mainly composed of three parts, which are the mean square error, sparsity penalty, and weight attenuation. The mean square error describes the difference between the observed value and the expected value. Given a data set (*a*^*m*^, *b*^*m*^) with *m* training samples, where *a*^*i*^ represents a piece of input data and *J* represents its label, the mean square error of the data sample is (*a*^*i*^, *b*^*i*^). It is defined as equation (15):

(15) $$\begin{array}{c} J\left(W,b,a,b\right)=\frac{1}{2}{\left\|h_{w,b}\left(a^{i}\right)-b^{i}\right\|}^{2}. \end{array}$$

Therefore, the number of hidden layer nodes that the entire neural network activates in each training is limited. Use *x*_*j*_^2^(*a*^*i*^) to represent the output of the *j*-th node when the input data is *a*^*i*^ in the second layer of the network, as in formula (16):

(16) $$\begin{array}{c} \rho_{j}=\frac{1}{m}\overset{m}{\underset{i=1}{\sum }}x_{j}^{2}\left(a^{i}\right). \end{array}$$

*x*_*j*_^2^ represents the impact of the output of this point on all *m* samples, that is, the average activation value. In addition, the sparsity parameter *ρ* in the sparsity penalty is generally set to a value slightly greater than but very close to 0 to ensure that the entire network is sparse.

Finally, in order to prevent the problem of over-fitting in this network, a weight attenuation term must be added. The weight attenuation term controls the entire network structure by reducing the range of weights and prevents overfitting to the input data. The weight attenuation parameter can describe the effect of this term in the cost function. If *J*_*wd*_ is too small, the weight attenuation term *J*_*wd*_ has too little influence on the cost function ∑_*i*=1_^*n*_*j*_−1^(*w*_*ji*_^*i*^)^2^, and fitting is prone to occur. The weight attenuation term is as shown in formula (17):

(17) $$\begin{array}{c} J_{wd}=\frac{\lambda }{2}\overset{n_{j}-1}{\underset{i=1}{\sum }}{\left(w_{ji}^{i}\right)}^{2}. \end{array}$$

Backpropagation algorithm is a supervised learning method, which can adjust the parameters of the entire network by comparing the difference between the expected value (*W*, *b*) and the real output *λW*_*ij*_^*i*^. The gradient formula *δ*/*δw*_*ij*_^*i*^ is as in formula (18):

(18) $$\begin{array}{c} \frac{\delta }{\delta w_{ij}^{i}}J_{Spaese}\left(W,b\right)=\frac{1}{m}\overset{m}{\underset{i=1}{\sum }}\frac{\delta }{\delta w_{ij}^{i}}+\lambda W_{ij}^{i}. \end{array}$$

In the training process of the neural network model, the error can also be transmitted through the backpropagation algorithm. The error of the last layer is as shown in formula (19):

(19) $$\begin{array}{c} \delta_{i}^{ni}=\frac{\delta }{\delta z_{i}^{ni}}\frac{1}{2}{\left\|b-h_{w,b}\left(a\right)\right\|}^{2}. \end{array}$$

In the forward propagation process, the error of the *l*-th layer can be calculated by the error of the latter layer, that is, the *l* + 1-th layer. The error calculation formula of the first layer is as formula (20):

(20) $$\begin{array}{c} \delta_{i}^{l}=\overset{s_{i+1}}{\underset{j=1}{\sum }}W_{ji}^{l}\delta^{l+1}+\beta {\left(-\frac{\rho }{1-\rho }\right)}^{2}. \end{array}$$

After obtaining the cost function, gradient, and error expression and transfer method, the algorithm can be used to train the entire network. First, train the network of each layer separately and then use the output of each layer as the network input of the next layer to complete the pretraining process of the entire neural network model.

## 5. Experiment and Analysis of the Harm of Parkinson's Disease and the Curative Effect of Moxibustion on Parkinson's Disease

### 5.1. Experiment and Analysis of the Harm of Parkinson's Disease

In recent years, the research on the nonmotor symptoms of Parkinson's disease has attracted more and more attention from clinicians. The general symptoms of Parkinson's disease are mainly divided into four main aspects: autonomic nerve dysfunction, neuropsychiatric disorders, sensory disorders, and sleep disorders. It can also cause the patient's motor symptoms to worsen. Seriously affect the quality of life of patients and their families, and may even shorten the life of patients. Therefore, timely detection and diagnosis of Parkinson's disease and reasonable implementation of treatment strategies have a great impact on improving the efficacy and quality of life of patients with Parkinson's disease.

This article investigates and analyzes the harm caused by Parkinson's disease, as shown in Figure 8.

As shown in Figure 8, Parkinson's disease is a neurological disease that often occurs in middle-aged and elderly people. Delays in action may also cause depression, mental disorders, negative attitudes towards life, and even dementia in the elderly. Elderly people should be actively treated and recuperated after discovering Parkinson's disease. With the increase of age, the chances of middle-aged and elderly people suffering from diseases are getting higher and higher. Many elderly people may suffer from Parkinson's disease. Parkinson's disease will also have a great impact on the lives of the elderly and their families.

This article investigates the development trend of Parkinson's disease from 2016 to 2020, as shown in Table 1.

As shown in Table 1, in 2016, there were 56743 people suffering from Parkinson's disease, accounting for 15%, and the growth rate was 5%; in 2017, there were 67,868 people suffering from Parkinson's disease, accounting for 18. %, the growth rate is 3%; the number of people suffering from Parkinson's disease in 2018 is 89,074, accounting for 22%, and the growth rate is 4%; the number of people suffering from Parkinson's disease in 2020 is 123,420 people, the percentage is 38%, and the growth rate is 9%. It can be seen that the number of people suffering from Parkinson's disease is increasing, the proportion is increasing, and the growth rate is increasing.

This article investigates the prevalence of Parkinson's disease by surveying 100 people of different age ranges, as shown in Table 2.

As shown in Table 2, divide 100 people into 4 different age ranges, and the number of people in each age range is the same. A survey of people in these four different areas found that only people aged 40-55 and 55-70 suffer from Parkinson's disease. Among the 25 survey subjects aged 55-70, 5 suffer from Parkinson's disease. It shows that people with Parkinson's disease are all older.

This article conducted a survey of these 6 patients on their own situation, as shown in Table 3.

As shown in Table 3, through the investigation of 6 patients with history of Parkinson's disease, it can be found that only 2 patients have a history of genetic disease, indicating that Parkinson's disease is not very related to the history of genetic disease. Only one patient had heart disease, indicating that Parkinson's disease and heart disease have little to do with each other.

### 5.2. Experiment and Analysis of the Curative Effect of Moxibustion on Parkinson's Disease

With the in-depth understanding of modern Chinese medicine and moxibustion treatment experience, more scientific dialectics and treatment methods have gradually formed. This study analyzes the hazards of Parkinson's disease patients through a clear diagnosis, investigates the main clinical characteristics of Parkinson's disease patients, and provides a reference basis for moxibustion treatment.

This article investigates the effects of moxibustion on people, as shown in Figure 9.

As shown in Figure 9, moxibustion is one of the most commonly used treatment methods in traditional Chinese medicine. Moxibustion can not only warm the meridians and relieve cold, promote qi and dredge the collaterals, strengthen the body, detoxify and relieve heat, eliminate blood stasis and cold, etc., but it is also used in health care. The effect of moxibustion on warming the meridian and dispelling cold reached more than 7 points, the effect on promoting qi and dredging collaterals reached more than 6.5 points, and the effect on strengthening the body reached an average of more than 7 points. Moxibustion is an area of traditional Chinese medicine, because moxibustion burning can stimulate acupuncture points. With the advancement of modern technology and the gradual improvement of people's health awareness, moxibustion as a natural remedy has received great attention.

This article investigates the efficacy of Western medicine and moxibustion on Parkinson's disease, as shown in Tables 4 and 5.

As shown in Tables 4 and 5, through the investigation and comparison of the two groups of patients with Western medicine treatment and moxibustion treatment, it can be found that the effect of Western medicine treatment is actually similar to that of patients using moxibustion, and the treatment time is about 60 days. The curative effect of patients using Western medicine treatment is about 34% on average, and the improvement of patients' quality of life is 56% on average; the curative effect of patients using moxibustion is about 40% on average, and the improvement of patients' quality of life is on average 65%. Both methods have improved the quality of life of patients, but the effect is not very obvious. However, the effect of moxibustion treatment on patients is slightly better than that of Western medicine treatment, but it has not achieved the desired effect.

Therefore, from the perspective of motor function, it is found that moxibustion may be an effective treatment method to improve Parkinson's disease, but it still needs more and more high-quality moxibustion to support. In addition, in clinical application, moxibustion can be divided into moxibustion moxibustion, grain moxibustion, etc. The specific method selection needs further research. Moxibustion can delay and improve the related symptoms of Parkinson's disease.

But moxibustion alone is less effective in treating Parkinson's disease. Moxibustion belongs to Chinese medicine and has the functions of strengthening, nourishing, and relieving muscle tension. Moxibustion treatment for patients with Parkinson's disease who are slow in movement or lack of energy has a certain effect on relieving symptoms. But moxibustion alone cannot control the overall progression of Parkinson's disease. So this article combines moxibustion with Western medicine.

A meta-analysis generally uses a funnel chart and judges whether there is a publication bias by whether the funnel chart is symmetric. When there is publication bias, it is manifested as an asymmetry in the funnel graph and a skewed distribution. This article compares the treatment with moxibustion and moxibustion combined with Western medicine, as shown in Figure 10.

As shown in Figure 10, moxibustion combined with Western medical treatment can effectively improve the motor symptoms of Parkinson's disease patients. The curative effect of moxibustion alone is between 40% and 50%, while the curative effect of moxibustion combined with Western medicine has reached more than 80%. The mechanism may be related to the etiology of Parkinson's disease. Compared with single Western medicine therapy, moxibustion combined with Western medicine therapy may have advantages in improving motor function analysis.

## 6. Discussion

This article analyzes how to study whether moxibustion therapy has an effect on the efficacy of Parkinson's disease based on smart medicine. Explain the related concepts of smart medicine and meta-analysis, and study the deep learning based on smart medicine. Explains the relevant theoretical knowledge of deep learning, explores the methods of deep learning research, and discusses whether moxibustion is feasible for the treatment of Parkinson's disease through experiments and analysis of various algorithms. Finally, it is integrated into the treatment of Parkinson's disease. Meta-analysis and moxibustion treatment are taken as examples to analyze.

This article also makes reasonable use of deep learning algorithms based on intelligent medical care. As the scope of deep learning applications becomes larger and larger, and its importance increases, many scholars have begun to apply deep learning to all aspects of life. According to this algorithm, it is known that moxibustion has a very good effect in the curative effect of moxibustion in the treatment of Parkinson's disease.

Through experimental analysis, this article knows that with the increasing growth rate of Parkinson's disease in recent years, the pace of research on the treatment of Parkinson's disease should also be accelerated. Experiments have found that moxibustion can effectively improve some of Parkinson's disease. Symptoms can help Parkinson's disease patients to reduce the harm such as slow movement. However, a single moxibustion treatment is not as effective as a combination of moxibustion and Western medicine. Therefore, a combination of moxibustion and Western medicine should be used to improve the symptoms of Parkinson's disease patients.

## 7. Conclusions

This article mainly discusses the research on the efficacy of moxibustion in the treatment of Parkinson's disease based on the meta-analysis of smart medical care. Intelligent medical treatment proposes a deep learning method. Deep learning method plays a huge role in intelligent medical care, so this method is adopted in this article. The method partly based on deep learning proposed algorithms such as convolutional neural network, restricted Boltzmann machine, and cost function. These algorithms are widely used in life, as well as in medicine. The experimental part of the experimental analysis of Parkinson's disease found that in recent years, the prevalence of Parkinson's disease in middle-aged and elderly people is increasing year by year. Therefore, research on the treatment of Parkinson's disease is currently the most important issue. Through the analysis of the harm caused by Parkinson's disease, it is found that it will bring many harms to patients, such as Alzheimer's disease, slow movement, and reduced quality of life. Finally, through experimental analysis of the role of moxibustion in the efficacy of Parkinson's disease, it is found that although a single moxibustion treatment can also improve the symptoms of Parkinson's disease, the combination of moxibustion and Western medicine has a better effect. Therefore, a combination of moxibustion and Western medicine should be used to treat patients with Parkinson's disease. This brings important significance to Parkinson's disease.

## Figures and Tables

**Figure 1:** Symptoms of PD patients.

**Figure 2:** Smart medical system structure.

**Figure 3:** Application of moxibustion.

**Figure 4:** Multifunctional intelligent moxibustion device.

**Figure 5:** System structure diagram of a meta-analysis.

**Figure 6:** Deep learning structure diagram.

**Figure 7:** Convolutional neural network structure diagram.

**Figure 8:** Harm caused by Parkinson's disease.

**Figure 9:** The effects of moxibustion.

**Figure 10:** Comparison of moxibustion and moxibustion combined with Western medicine.

**Table 1:** Development trend of Parkinson's disease from 2016 to 2020.

Years	Case	Percentage	Growth rate
2016	56743	15%	5%
2017	67868	18%	3%
2018	89074	22%	4%
2019	90750	29%	7%
2020	123420	38%	9%

**Table 2:** Probability of Parkinson's disease in different age ranges.

Age range	Total people	Number of patients	Percentage	Effective percentage
10-25	25	0	0	0
25-40	25	0	0	0
40-55	25	1	1%	1%
55-70	25	5	5%	5%

**Table 3:** 6 investigations of patients' own situation.

Survey object	Genetic history	Sporadic cases	Heart disease	Percentage
1	Yes	No	No	16%
2	No	No	No	0
3	No	No	No	0
4	Yes	No	No	16%
5	No	No	No	0
6	No	No	Yes	0

**Table 4:** Efficacy of Western medicine on Parkinson's disease.

Survey object	Treatment time (days)	Curative effect	Quality of life
A	60	35%	58%
B	65	33%	55%
C	67	32%	54%
D	63	36%	56%
E	66	37%	56%

**Table 5:** Efficacy of moxibustion on Parkinson's disease.

Survey object	Treatment time (days)	Curative effect	Quality of life
A	60	39%	65%
B	65	38%	67%
C	67	42%	64%
D	63	43%	63%
E	66	46%	66%

## Data Availability

The data that support the findings of this study are available from the corresponding author upon reasonable request.
